RETRACTED

# Different Scores Predict the Value of Hemorrhagic Transformation after Intravenous Thrombolysis in Patients with Acute Ischemic Stroke

**DOI:** 10.1155/2021/2468052

**Published:** 2021-10-21

**Authors:** Xiaozan Chang, Xiaoxi Zhang, Guanglin Zhang

**Affiliations:** ^1^Neurosurgery Department of Stroke Center, Henan Provincial People's Hospital, Zhengzhou, China; ^2^Cerebrovascular Department of Interventional Center, Zhengzhou University People's Hospital, Zhengzhou, China; ^3^Stroke Center, Naval Medical University First Affiliated Hospital, Shanghai 200433, China

## Abstract

**Objective:**

To evaluate the value of the Alberta stroke project early CT score (ASPECTS), DRAGON score, SEDAN score, and HAT score in predicting hemorrhagic transformation (HT) after intravenous thrombolysis in patients with acute ischemic stroke (AIS).

**Methods:**

The clinical data of 248 AIS patients treated with intravenous thrombolysis in our hospital from December 2017 to December 2019 were analyzed. According to the prognosis, all patients were divided into the non-HT group (*n* = 200) and the HT group (*n* = 48). Univariate analysis and multivariate logistic regression models were used to analyze clinical data to determine the influencing factors of HT after intravenous thrombolysis in AIS patients. The receiver operating characteristic curve was used to evaluate the ASPECTS, DRAGON, SEDAN, and HAT scores to the value of predicting HT after intravenous thrombolysis in AIS patients.

**Results:**

The lower the ASPECTS score and the higher the DRAGON, SEDAN, and HAT scores, the higher the incidence of HT after intravenous thrombolysis in AIS patients (*P* < 0.05). The results of multivariate logistic regression analysis showed that the patient's age, atrial fibrillation, baseline NIHSS score, early signs of infarction on admission with head CT, time from onset to thrombolytic therapy, and thrombolytic drugs were all independent factors affecting intravenous thrombolysis in AIS patients (*P* < 0.05). The area under the curve (AUC) of the predictive value of ASPECTS for HT is 0.895 (95% CI 0.813–0.977). When the optimal cutoff value is 0.607, the sensitivity is 100% and the specificity is 60.7%. The AUC of the predictive value of DRAGON for HT is 0.877 (95% CI 0.790–0.964). When the optimal cutoff value is 0.665, the sensitivity is 84.4% and the specificity is 82.1%. The AUC of the predictive value of SEDAN for HT is 0.764 (95% CI 0.638–0.890). When the optimal cutoff value is 0.474, the sensitivity is 78.6% and the specificity is 68.8%. The AUC of the predictive value of HAT for HT is 0.777 (95% CI 0.651–0.903). When the optimal cutoff value is 0.509, the sensitivity is 68.8% and the specificity is 82.1%.

RETRACTED

**Conclusion:**

The lower the ASPECTS score and the higher the DRAGON, SEDAN, and HAT scores, the higher the incidence of HT in AIS patients. The patient's age, atrial fibrillation, baseline NIHSS score, early signs of infarction on admission with head CT, time from onset to thrombolytic therapy, and thrombolytic drugs are all independent factors affecting HT in AIS patients. The scores of ASPECTS, DRAGON, SEDAN and HAT have certain value in predicting HT after intravenous thrombolysis in AIS patients, and the predicted value of ASPECTS score is the best.

## 1. Introduction

Acute ischemic stroke (AIS) refers to a kind of clinical syndrome in which the cerebral blood supply disorder caused by various cerebrovascular diseases leads to local brain tissue ischemia and hypoxic necrosis and the rapid appearance of corresponding neurological deficits [1]. At present, the treatment of AIS mainly includes intravenous thrombolysis, vascular intervention, and anticoagulant therapy. Among them, intravenous thrombolysis is currently the most important measure to restore blood flow, and recombinant tissue plasminogen activator (rt-PA) and urokinase are the main thrombolytic drugs currently used in China [2]. Intravenous thrombolysis is designed to reduce and relieve brain tissue ischemia by rapidly recanalizing occlusive blood vessels, thus maximizing the recovery of its nerve function. However, in the process of intravenous thrombolysis therapy, there will be the low vascular recanalization rate, intracranial hemorrhage transformation (HT), ischemia/reperfusion injury, vascular reocclusion, and so forth, which will affect the prognosis of patients [3]. It is crucial to predict early and timely HT in AIS patients after intravenous thrombolysis and improve the efficacy of intravenous thrombolysis to reduce the mortality of patients. So finding a simple and effective clinical evaluation method has become the key content to predict HT. Alberta stroke project early CT score (ASPECTS) can visually evaluate the ischemia of the brain tissue of AIS patients by obtaining the information of the ischemic location of the brain tissue [4]. The DRAGON score is based on the variables available for AIS patients before admission to treatment and integrates the patient's clinical characteristics, laboratory tests, and imaging information [5]. The SEDAN score, widely used in clinic, involves few variables and is convenient and practical [6]. The hemorrhage after thrombolysis (HAT) score is a neuropsychological measurement scale, which contains three simple indicators and can rapidly predict the prognosis of AIS patients [7]. This study explored the risk factors of HT after intravenous thrombolysis in AIS patients and compared the predictive value of different scales for HT in order to provide reference for the treatment of AIS patients. The specific report is as follows.

RETRACTED

## 2. Subject and Methods

### 2.1. Subject

The clinical data of 248 AIS patients treated with rt-PA intravenous thrombolysis in our hospital from December 2017 to December 2019 were collected retrospectively. Inclusion criteria were as follows: all patients met the diagnostic criteria of “European Stroke Organisation (ESO) guidelines for prophylaxis for venous thromboembolism in immobile patients with acute ischemic stroke [8],” and intravenous thrombolysis with rt-PA was performed within 4.5 hours of onset or with urokinase within 6 hours of onset. According to the prognosis, the patients were divided into the non-HT group (*n* = 200) and HT group (*n* = 48).

### 2.2. Methods

The study collected patient gender, age, body weight, past history (including hypertension, diabetes, cerebral infarction, coronary heart disease, atrial fibrillation, smoking, and alcohol consumption), baseline indicators (including baseline National Institutes of Health Stroke Scale (NIHSS), baseline systolic blood pressure, and baseline blood glucose), early infarction signs on admission with head CT, the time from onset to thrombolytic therapy, and so forth.

All patients were treated with intravenous thrombolytic therapy of rt-PA or urokinase after onset. rt-PA 0.9 mg/kg (maximum dose 90 mg) was given by intravenous drip, of which 10% was given by venous pushing injection within the first 1 min and the rest was instilled continuously for 1h. Urokinase, 1,000,000–1,500,000 IU, dissolved in 100–200 ml normal saline, was given by continuous intravenous drip for 30 min. During intravenous thrombolysis and within 24 hours of medication, the patients were closely monitored, and blood pressure and neurological function were measured regularly.

The ASPECTS, DRAGON, SEDAN, and HAT scores were used for measurement, and all patients were evaluated by the scale after intravenous thrombolysis and medication for 24 hours. ASPECTS is to used to evaluate the area of cerebral ischemia by selecting 10 brain tissue sites. Within 6 hours of the onset of HT, the CT scan of the brain tissue showed low-density shadows. If the 10 sites included in the ASPECTS were involved, then the number of brain tissue sites involved was subtracted from the total score. The higher the ASPECTS, the lower the incidence of HT after intravenous thrombolysis in AIS patients. DRAGON score included age, blood sugar, and other variables. The higher the DRAGON, the higher the incidence of HT after intravenous thrombolysis in AIS patients. SEDAN includes blood glucose, CT signs of ischemia in the early stage of onset, and other variables; its total score is 6 points, and the higher SEDAN, the higher the incidence of HT in AIS patients after intravenous thrombolysis. The HAT score included NIHSS, age, diabetes, and other variables, and the total score was 5. The higher the HAT score, the higher the incidence of HT in AIS patients after intravenous thrombolysis.

RETRACTED

### 2.3. Statistical Analysis

Data were processed by the SPSS 22.0. The enumeration data is expressed by percentage (%). Multigroup comparison of quantitative data between groups was performed by analysis of variance, and the *t*-test was used for pairwise comparison. The chi-square test was used for the enumeration data. The influencing factors of patients were analyzed by multivariate logistic regression analysis. Meanwhile, receiver operating characteristic curve (ROC) was drawn, and the area under the ROC curve (AUC) was used to evaluate the prediction of HT after AIS intravenous thrombolysis by ASPECTS, DRAGON, SEDAN, and HAT scores. Differences were considered statistically significant at *P* < 0.05.

## 3. Results

### 3.1. Four Types of Scores for Patients

The lower the ASPECTS score, the higher the DRAGON, SEDAN, and HAT scores and the higher the incidence of HT after intravenous thrombolysis in AIS patients. The differences were statistically significant (*P* < 0.05), as shown in Table 1.

### 3.2. Univariate Analysis of HT after Intravenous Thrombolysis in AIS Patients

Univariate analysis showed that age, atrial fibrillation, baseline NIHSS score, baseline blood glucose, early signs of infarction on admission with head CT, time from onset to thrombolytic therapy, and thrombolytic drugs were all closely related to the occurrence of HT after intravenous thrombolysis in AIS patients, with statistically significant differences (*P* < 0.05), as shown in Table 2.

### 3.3. Multivariate Logistic Regression Analysis of HT in AIS Patients after Intravenous Thrombolysis

The results of multivariate logistic regression analysis showed that age, atrial fibrillation, baseline NIHSS, early infarction signs on admission with head CT, time from onset to thrombolytic therapy, and thrombolytic drugs were all independent influencing factors of intravenous thrombolysis in AIS patients, and the differences were all statistically significant (*P* < 0.05), as shown in Tables 3 and 4.

### 3.4. The Value of Four Scoring Methods in Predicting HT after Intravenous Thrombolysis in AIS Patients

The area under the curve (AUC) of the predictive value of ASPECTS for HT after intravenous thrombolysis in AIS patients is 0.895 (95% CI 0.813–0.977). When the optimal cutoff value is 0.607, the sensitivity is 100% and the specificity is 60.7%. The AUC of the predictive value of DRAGON for HT after intravenous thrombolysis in AIS patients is 0.877 (95% CI 0.790–0.964). When the optimal cutoff value is 0.665, the sensitivity is 84.4% and the specificity is 82.1%. The AUC of the predictive value of SEDAN for HT after intravenous thrombolysis in AIS patients is 0.764 (95% CI 0.638–0.890). When the optimal cutoff value is 0.474, the sensitivity is 78.6% and the specificity is 68.8%. The AUC of the predictive value of HAT for HT after intravenous thrombolysis in AIS patients is 0.777 (95% CI 0.651–0.903). When the optimal cutoff value is 0.509, the sensitivity is 68.8% and the specificity is 82.1%, as shown in Table 5 and Figure 1.

RETRACTED

## 4. Discussion

AIS is a disease with rapid localized or diffuse brain function impairment caused by cerebrovascular stenosis or occlusion, and corresponding abnormal signs of nervous system such as limb paralysis, sensory impairment, and speech dysfunction often occur [9]. For AIS patients, blocked blood vessels should be opened as soon as possible to restore blood perfusion and promote nerve recovery. Active restoration of vascular recanalization will increase the risk of HT, seriously affect the recovery of patients' neurological function, and lead to disability or even death [10, 11]. Therefore, how to predict the risk of HT in AIS patients after intravenous thrombolytic therapy and improve the efficacy and safety of thrombolytic therapy has become an important issue facing clinicians.

The scales of ASPECTS, DRAGON, SEDAN, and HAT can all predict the occurrence of HT after intravenous thrombolysis in AIS patients. The ASPECTS is a simple, reliable, and systematic scoring system. Prognosis of anterior circulation and posterior circulation in AIS patients after intravenous thrombolysis can be accurately predicted by the ASPECTS within 6 h of acute onset [12]. DRAGON score is a scoring system based on patients with anterior circulation, which makes rapid evaluation and accurate judgment of patients' conditions with reference to patients' age, baseline blood glucose level, NISHH score, time from onset to treatment, and other results [13]. SEDAN score is a practical scoring system involving fewer variables, which can predict HT after intravenous thrombolysis in AIS patients [14]. HAT is a simple and easy-to-operate neuropsychological measurement scale that can make basic judgments on the prognosis of AIS patients. In conclusion, it is of great significance to find a simple and feasible method to assess the risk of HT in AIS patients after intravenous thrombolysis.

RETRACTED

The results of this study showed that the lower ASPECTS and the higher DRAGON, SEDAN, and HAT scores, the higher the incidence of HT in AIS patients after intravenous thrombolysis. The reason is that ASPECTS was used to score patients with AIS based on the bleeding of 10 sites of brain tissues, and the number and degree of bleeding sites were closely related to the occurrence of HT in AIS patients, so the higher the ASPECTS and the lower the incidence of HT in AIS patients after thrombolytic therapy. DRAGON, SEDAN, and HAT scores are used to judge the condition of AIS patients; the higher the scores of them, the more severe the patient's condition and the higher the incidence of HT in AIS patients after thrombolytic treatment.

The results of this study showed that patients' age, atrial fibrillation, baseline NIHSS, baseline blood glucose, early infarction signs on admission with head CT, time from onset to thrombolytic therapy, and thrombolytic drugs were closely related to the occurrence of HT in AIS patients after intravenous thrombolytic therapy. Among them, patients' age, atrial fibrillation, baseline NIHSS, early infarction signs on admission with head CT, time from onset to thrombolytic therapy, and thrombolytic drugs were all independent influencing factors of HT in AIS patients after intravenous thrombolytic therapy. The reason is that the prognosis of patients (>65 years old) with intravenous thrombolytic therapy is worse than that of younger patients, which is the relative contraindication of intravenous thrombolysis. Patients with a history of atrial fibrillation can aggravate the condition of cardiogenic cerebral embolism, resulting in that the risk of intracranial hemorrhage after thrombolysis is higher [15, 16]. Baseline NIHSS can reflect the severity of the disease, and the higher the baseline NIHSS, the more severe the disease. Head CT signs can show the range of infarction or hemorrhage in AIS patients. The larger the lesion area of AIS is, the higher the degree of tissue ischemia is, and the more likely it is to develop HT after thrombolysis in AIS patients [17]. Within 3 h of onset, rt-PA standard intravenous thrombolytic therapy is the only treatment method for AIS that has been proved to have significant efficacy by rigorous clinical scientific experiments and has been approved for clinical application. If rt-PA is used unconditionally and within 6 h of onset, patients can also receive intravenous thrombolytic therapy through urokinase. The use of rt-PA within 3 h of the onset can effectively reduce the occurrence of postoperative HT [18].

The ROC curve results showed that AUC of HT predicted by ASPECTS, DRAGON, SEDAN, and HAT scores after intravenous thrombolysis in AIS patients were 0.895, 0.877, 0.764, and 0.777, respectively. The results showed that ASPECTS, DRAGON, SEDAN, and HAT scores had certain value in predicting HT after intravenous thrombolysis in AIS patients, and, among them, ASPECTS scale has the highest predictive value for the occurrence of HT in AIS patients, while SEDAN scale has the lowest predictive value. The reason is that ASPECTS can be used to assesses the number of ischemic sites in brain tissue, so as to intuitively and clearly obtain the size of ischemic sites and the severity of cerebral ischemia, which has been widely used to assess intravenous thrombolytic finger syndrome [19]. The indicators of DRAGON are few and can be obtained before treatment, which is highly practical and widely used in clinical practice. SEDAN is a simple and practical assessment method, including patients' age, blood glucose, cranial CT, and other indicators, which are easy to obtain and can be used to predict the risk of postcirculation HT. HAT score has three indicators: blood glucose, NISHH, and cranial CT, which can rapidly predict the prognosis of AIS patients [20]. Therefore, when AIS patients have risk factors for HT, the corresponding scale should be used for evaluation when intravenous thrombolysis is performed according to the patient's condition characteristics, so as to prevent and intervene in the occurrence of HT as early as possible. Besides, ASPECTS is the most recommended scale for evaluation, while SEDAN scale has poor applicability.

RETRACTED

## 5. Conclusion

The patients' age, atrial fibrillation, baseline NIHSS score, early signs of infarction on admission with head CT, time from onset to thrombolytic therapy, and thrombolytic drugs are all independent factors affecting intravenous thrombolysis in AIS patients. ASPECTS, DRAGON, SEDAN, HAT, and other scores predict the value of HT after AIS intravenous thrombolysis. Among them, the predicted value of ASPECTS score is the largest.

## Figures and Tables

**Figure 1:** The ROC curve of four scoring methods in predicting HT after intravenous thrombolysis in AIS patients. Note: when the ROC curve was close to or below the standard line, it represented the low authenticity of the test method, while when it was closer to the upper left of the ROC curve, it represented the high authenticity of the test method, which had good application value.

**Table 1:** Four types of scores for patients (*n*, %).

	No HT group (*n* = 200)	HT group (*n* = 48)			
		Asymptomatic hemorrhage	Symptomatic hemorrhage	Fatal hemorrhage	Total incidence rate
*ASPECTS (point)*					
0∼3 (*n* = 14)	6 (42.85%)	2 (14.29%)	3 (21.43%)	3 (21.43%)	8 (57.15%)
4∼6 (*n* = 60)	44 (73.33%)	10 (16.67%)	5 (8.33%)	1 (1.67%)	16 (26.67%)^*∗*^
7∼8 (*n* = 88)	74 (84.09%)	10 (11.36%)	4 (4.55%)	0 (0%)	14 (15.91%)^*∗*^^#^
9∼10 (*n* = 86)	76 (88.37%)	9 (10.47%)	1 (1.16%)	0 (0%)	10 (11.63%)^*∗*^^#△^
*χ* ^*2*^ *value*					18.822
*P* value					＜0.001

*DRAGON score (point)*					
0∼4 (*n* = 90)	86 (95.56%)	4 (4.44%)	0 (0%)	0 (0%)	4 (4.44%)
5∼9 (*n* = 66)	61 (92.42%)	4 (6.10%)	1 (1.52%)	0 (0%)	5 (7.58%)^*∗*^
10∼15 (*n* = 51)	36 (70.59%)	8 (15.68%)	6 (11.76%)	1 (1.96%)	15 (29.41%)^*∗*^^#^
＞15 (*n* = 41)	17 (41.46%)	15 (36.59%)	6 (14.63%)	3 (7.32%)	24 (58.53%)^*∗*^^#△^
*χ* ^*2*^ value					62.316
*P* value					＜0.001

*SEDAN score (point)*					
0 (*n* = 51)	49 (96.08%)	2 (3.92%)	0 (0%)	0 (0%)	2 (3.92%)
1 (*n* = 90)	76 (84.44%)	10 (11.11%)	3 (3.33%)	1 (1.11%)	14 (15.56%)^*∗*^
2 (*n* = 60)	45 (75.00%)	10 (16.67%)	4 (26.67%)	1 (1.67%)	15 (25.00%)^*∗*^#
3–6 (*n* = 47)	30 (63.83%)	9 (19.15%)	6 (12.77%)	2 (4.26%)	17 (36.17%)^*∗*^#△
*χ* ^2^ value					18.354
*P* value					<0.001

*HAT score (point)*					
0 (*n* = 108)	96 (88.89%)	11 (10.19%)	1 (0.93%)	0 (0%)	12 (11.11%)
1 (*n* = 68)	60 (88.24%)	7 (10.29%)	1 (1.47%)	0 (0%)	8 (11.76%)^*∗*^
2 (*n* = 37)	27 (72.97%)	5 (13.51%)	4 (10.81%)	1 (2.70%)	10 (27.03%)^*∗*^#
3–5 (*n* = 35)	17 (48.57%)	8 (22.86%)	7 (20.00%)	3 (8.57%)	18 (51.43%)^*∗*^#△
*χ* ^*2*^ *value*					31.675
*P* value					＜0.001

Comparison with 0–3 points, ^*∗*^*P* < 0.05; comparison with 4–6 points, #*P* < 0.05; comparison with 7–8 points, △*P* < 0.05; comparison with 0–4 points, ^*∗*^*P* < 0.05; comparison with 5–9 points, #*P* < 0.05; comparison with 10–15 points, △*P* < 0.05; comparison with 0 points, ^*∗*^*P* < 0.05; comparison with 1 point, #*P* < 0.05; comparison with 2 points, △*P* < 0.05; comparison with 0 points, ^*∗*^*P* < 0.05; comparison with 1 point, #*P* < 0.05; comparison with 2 points, △*P* < 0.05.

RETRACTED

**Table 2:** Univariate analysis of HT after intravenous thrombolysis in AIS patients (*n*, %).

Factors		No HT group (*n* = 200)	HT group (*n* = 48)	*χ* ^2^ value	*P* value
Gender	Male	145	35	1.003	0.954
	Female	55	13		

Age (years)	≤65	97	33	6.364	0.012
	>65	103	15		

Weight (kg)	≤70	88	23	0.240	0.624
	>70	122	25		

History of hypertension	Yes	113	23	1.152	0.283
	No	87	25		

History of diabetes	Yes	98	20	0.835	0.361
	No	102	28		

History of cerebral infarction	Yes	91	27	1.794	0.080
	No	109	21		

History of coronary heart disease	Yes	79	26	3.411	0.065
	No	121	22		

Atrial fibrillation	Yes	84	30	6.550	0.010
	No	116	18		

Smoking history	Yes	85	27	2.956	0.086
	No	115	21		

Drinking history	Yes	121	25	1.133	0.287
	No	79	23		

Baseline NIHSS score (point)	≤14	102	15	6.059	0.014
	>14	98	33		

Baseline systolic pressure (mmHg)	≤155	90	15	2.998	0.083
	>155	110	33		

Baseline blood glucose (mmol/L)	≤7.8	119	18	7.578	0.006
	>7.8	81	30		

Early signs of infarction on admission with head CT	Yes	99	32	4.578	0.032
	No	101	16		

Time from onset to thrombolytic therapy (h)	≤3	90	8	13.002	≤0.01
	>3, and ≤4.5	110	40		

Thrombolytic drugs	rt-PA	98	12	9.034	0.003
	Urokinase	102	36		

**Table 3:** Assignment value of multivariate analysis.

Factors	Assignment value
Age (years)	“≤ 65” = “0”; “> 65” = “1”
Atrial fibrillation	“No” = “0”; “yes” = “1”
Baseline NIHSS score (point)	“≤ 14” = “0”; “> 14” = “1”
Baseline blood glucose (mmol/L)	“≤ 7.8” = “0”; “> 7.8” = “1”
Early signs of infarction on admission with head CT	“No” = “0”; “yes” = “1”
Time from onset to thrombolytic therapy(h)	“≤ 3” = “0”; “> 3, and ≤4.5” = “1”
Thrombolytic drugs	“rt-PA” = “0”; “yes” = “1”

**Table 4:** Multivariate logistic regression analysis of HT in AIS patients after intravenous thrombolysis.

Factors	B value	SE	Walds	OR value	95% CI	*P* value
Age	0.135	0.056	5.786	0.960	0.932–0.979	0.026
Atrial fibrillation	0.125	0.036	12.056	0.132	0.065–0.215	0.009
Baseline NIHSS score	0.298	0.124	5.768	0.331	0.128–0.792	0.033
Baseline blood glucose	0.146	0.081	3.244	0.948	0.908–0.981	0.125
Early signs of infarction on admission with head CT	0.356	0.121	8.650	0.905	0.802–1.013	0.011
Time from onset to thrombolytic therapy	0.452	0.166	7.414	0.425	0.119–0.688	0.028
Thrombolytic drugs	0.395	0.174	5.153	0.515	0.384–0.895	0.035

**Table 5:** Four scoring methods in predicting the value of HT after intravenous thrombolysis in AIS patients.

Scoring methods	AUC	Asymptotic 95% confidence interval		Optimal cutoff value	Sensitivity (%)	Specificity (%)
		Lower limit	Upper limit			
ASPECTS	0.895	0.813	0.977	0.607	100	60.7
DRAGON	0.877	0.790	0.964	0.665	84.4	82.1
SEDAN	0.764	0.638	0.890	0.474	78.6	68.8
HAT	0.777	0.651	0.903	0.509	68.8	82.1

## Data Availability

The data are available from the corresponding author upon request.
